# The mediating effects of hope on the relationships of social support and self-esteem with psychological resilience in patients with stroke

**DOI:** 10.1186/s12888-024-05744-w

**Published:** 2024-05-07

**Authors:** Boru Sun, Nan Wang, Ke Li, Yan Yang, Fengjiao Zhang

**Affiliations:** 1 Emergency Department, Shengjing Hospital of China Medical University, Shenyang, Liaoning China; 2 Rehabilitation Center, Shengjing Hospital of China Medical University, Shenyang, Liaoning China; 3 Surgery Department, Shengjing Hospital of China Medical University, Shenyang, Liaoning China; 4 Nursing Department, Shengjing Hospital China Medical University, 36 Sanhao Street, Heping District, Shenyang, Liaoning P.R. China; 5 Teaching Group of Nursing Department, Shengjing Hospital of China Medical University, 36 Sanhao Street, Heping District, Shenyang, Liaoning 110004 P.R. China

**Keywords:** Resilience, psychological, Social support, Self-concept, Hope, Stroke

## Abstract

**Purpose:**

To explore the mediating effect of hope in the relationships between social support and self-esteem with psychological resilience among patients with stroke survivors in early rehabilitation.

**Methods:**

A cross-sectional study design was adopted. Data from a cross-sectional survey of 210 patients undergoing early stroke rehabilitation were analyzed using structural equation modeling. The variables of interest were measured using the Connor Davidson Resilience Scale, the Social Support Rating Scale, the Herth Hope Index, and the Self-Esteem Scale. This article reports according to the STROBE checklist.

**Results:**

A positive relationship was found between social support and psychological resilience (*β*_*1*_ = 0.548), which was mediated by hope (*β*_*2*_ = 0.114), and social support had significant direct effect on resilience (*β*_*3*_ = 0.434). A positive relationship was also found between self-esteem and psychological resilience (*β*_*4*_ = 0.380), which was mediated by hope (*β*_*5*_ = 0.200), and self-esteem had significant direct effect on resilience (*β*_*6*_ = 0.179).

**Conclusion:**

According to the results of this study, some strategies can be incorporated into the rehabilitation process to enhance psychological resilience, such as cultivating individual personality characteristics and improving patients’ social relationships. In the future, we need to explore methods for improving psychological resilience among patients with stroke in combination with their risk factors to improve their quality of life and reduce the incidence of post-stroke depression.

**Supplementary Information:**

The online version contains supplementary material available at 10.1186/s12888-024-05744-w.

## Introduction

The significance of stroke is likely to increase in the future due to the aging populations in developing countries [1]. China has the highest lifelong risk of stroke worldwide [2], and one of the burdens is post-stroke depression, the most common non-cognitive neuropsychiatric complication of stroke [3], characterized by patients’ reduced participation in rehabilitation and increased rates of recurrence and mortality [4]. The evidence for specific therapies of stroke has been separated into two periods: early rehabilitation (< 6 months post-stroke) versus late rehabilitation (> 6 months post-stroke) treatment [5]. Post-stroke depression usually occurs within the first months after a stroke, then gradually increases, and eventually peaks within six months [6]. Therefore, methods to reduce the incidence of depression within 6 months (early rehabilitation) after stroke are important. A longitudinal study showed that resilience is a protective factor against post-stroke depression [7], and the rate of depression among patients with a high level of psychological resilience decreases over time. Resilience is defined as ‘the dynamic process of adapting well to trauma, adversity, threat, tragedy, or major sources of stress’ [8]. A positive outlook is an effective component of psychological resilience, which protects resilient people from depression and helps them obtain psychological resources [9]. Psychological resilience is also an independently related factor of quality of life in patients with first ischemic stroke [10]. A higher level of psychological resilience is related to a lower level of emotional distress and a higher quality of life [9]. From what is mentioned above, we can know that psychological resilience is an important outcome for stroke patients in early rehabilitation. Determining the key factors that affect the level of resilience after a stroke is important for planning and evaluating interventions for rehabilitation.

Hope, a dynamic and multi-level psychological process, is believed to be important in recovery and the perception of recovery from illness or injury. Qualitative and quantitative studies have shown that hope plays an important role in early post-stroke recovery [11–13] and is necessary for optimal recovery [14]. These studies have explored the important role of hope in post-stroke recovery, but have not explained the specific path of action.

## Psychological resilience

The psychological resilience of patients over the first 6 months following a first stroke is much worse than that of the general population [15, 16] and healthy older population [17]. Few conditions demand resilience more than stroke does [18]. Psychological resilience can greatly affect the recovery and adjustment process of patients with stroke, and it may be an important determinant of their future living arrangements. Changes in psychological resilience may be due to a combination of environmental and personal factors. Resilience is a continuous process, not necessarily a characteristic that a person has or does not have. For example, a person may cope very well in one situation but show low psychological resilience in another one [19]. Therefore, resilience has dynamic properties, and it can be learned and enhanced. A review summarized the factors that contribute significantly to psychological resilience, including biological factors (such as brain structure and function and neurobiological systems), personal factors (such as optimism, self-esteem, and hope), and environmental-systemic factors (such as social support) [20].

## Social support

Social support in this study refers to the spiritual and material help perceived, obtained, and used by patients with stroke, such as love and respect from others or groups, which can reduce stress. The research literature shows that a social support system is an important protective factor for individuals experiencing stressful events, and protective factors are necessary for the recovery process. Therefore, social support may be closely related to psychological resilience [21, 22]. Price et al. [23] found several prominent characteristics of stroke survivors with psychological resilience, one of which was the use of social support. Some researchers have developed group-based peer support interventions to improve the psychological resilience of patients with stroke, and the results have been positive [24]. However, few studies have been published on the relationship between psychological resilience and social support in convalescing patients with stroke; thus, it is necessary to further explore the relationship between them.

### Self-esteem

Self-esteem reflects people’s feelings about themselves and is a multifaceted construct related to other psychological constructs, such as self-image, self-concept, self-perception, self-confidence, self-acceptance, self-esteem, and self-worth [25]. For a long time, self-esteem has been a variable of interest in mental health research and has become an important variable in the health care. In recent years, the impact of self-esteem on stroke rehabilitation has received more attention in the literature with focusing on patients with acute stroke in the rehabilitation [26–29]. Self-esteem is considered to be an important factor affecting the emotional and functional outcomes of patients with chronic diseases (such as stroke) [28]. However, stroke survivors reported low self-esteem [30, 31]. Studies have explored the antecedents of self-esteem of stroke patients [32, 33), and others have shown that self-esteem and social support jointly affect the practice of self-care behaviour of stroke patients [34]. However, there is still a lack of research on the psychological impact of self-esteem after brain injury. People who have low self-esteem following acquired brain injury (including stroke) may be less able to utilize coping strategies and manage the physical, cognitive, psychological and psychosocial consequences of the injury if they are less able to focus on competence over limitations, or to maintain a sense of self-worth over feelings of hopelessness [35]. People with high self-esteem are more likely to attempt to increase their feelings of self-worth, whereas people with low or fragile self-esteem may be more unconsciously concerned with protecting the limited self-esteem resources they have, therefore becoming more reluctant to risk failure or rejection [36]. Therefore, we try to broaden our understanding of self-esteem by studying the impact of self-esteem on psychological resilience.

### Hope and its relationship with social support, self-esteem, and psychological resilience

Hope is a complex and multidimensional concept. Based on the findings of concept analysis, a multidimensional model of hope for people after stroke is proposed [37]. The key features depicted in the model include: (1) Hope being developed through a range of factors: internal (attitude, sense of self, previous experience), stroke-related (progress to date, severity), and external (family and friends, spiritual beliefs, staff); (2) Hope having 3 attributes - an inner state, an outcome-oriented attribute, and an active process; (3) Hope yielding positive outcomes that affect a person’s internal state (perseverance, motivation, coping, mood modulation) and recovery (increased participation, ongoing recovery, improved quality of life). There were 3 crucial factors in maintaining hope according to the model: a supportive environment (interconnectedness), a sense of belief in one’s self (positive attitude towards temporality and the future), and a belief that ongoing progress is possible (positive readiness and expectancy) [38].

Although hope can theoretically explain how social support and self-esteem affect patients’ psychological resilience after stroke, empirical studies are still in their infancy. Empirical studies from patients with other chronic diseases provided support for the relationship between these variables. Snyder’s theory of hope [39] shows that hope is a positive motivational state, which involves the evaluation of a person’s ability to achieve goals successfully, and may be affected by self-esteem. Specifically, self-esteem is an important motivator in the pursuit of self-worth. It can encourage individuals to use effective strategies to overcome difficulties, achieve goals, and have greater hope for the future [40]. Therefore, self-esteem is likely to play a positive role in improving hope. A narrative review [41] found that social support from friends and family members could be a potential factor in generating hope in stroke patients. In particular, social support can be a source of motivation and encouragement during the rehabilitation process, helping to foster or maintain a sense of hope among stroke survivors. A study on adolescents after an earthquake found that hope mediated social support and post-traumatic growth [42]. Snyder et al. suggested that social support could improve the level of personal hope by establishing and expanding personal resources [43]. In addition, the results of empirical research support the positive effect of social support on hope [44]. Therefore, we believe that social support can increase levels of psychological resilience among patients after stroke by increasing hope.

In summary, the first 6 months following a first stroke is the key period of rehabilitation, during which the patient’s psychological resilience plays an important role. In the multidimensional model of hope for people after stroke, psychological resilience is an important positive result of hope. This model explains the internal antecedents, external antecedents, and positive results of hope, but lacks the support of empirical research. Therefore, this study focused on internal antecedent - self-esteem, external antecedent - social support, and consequence - psychological resilience (Fig. 1). The aim of this study is to explore the mediating effect of hope in the relationships between social support and self-esteem with psychological resilience among patients with stroke survivors in early rehabilitation. Based on the above analysis and the multidimensional model of hope after stroke proposed by Bright et al. [38], the following research hypotheses are put forward:

**Fig. 1:** Hypothetic model

#### Hypothesis 1

Social support, hope and self-esteem of patients with stroke in early rehabilitation have a positive impact on their psychological resilience;

#### Hypothesis 2

Social support and self-esteem of patients with stroke in early rehabilitation have a positive impact on hope;

#### Hypothesis 3

The hope of patients with stroke in early rehabilitation is a mediator variable between social support and psychological resilience;

#### Hypothesis 4

The hope of patients with stroke in early rehabilitation is a mediator variable between self-esteem and psychological resilience.

## Methods

### Study design

A cross-sectional study design was used in this study.

### Settings, samples and data collection

This cross-sectional study was conducted from October 2020 to May 2021 in the rehabilitation center of a tertiary hospital in Liaoning Province. Due to the requirement of a sample size of at least 200 for structural equation modeling [45] and the principle that the sample size should be 10 times for each variable according to regression analysis [46], a total of 210 inpatients stroke patients were finally recruited by convenience sampling method to participate in the study.

The criteria for the inclusion of patients were as follows: (1) met the diagnostic criteria of the Chinese Society of Neurology and Chinese Stroke Society 2018; and were diagnosed with stroke using cranial CT, DSA or MRI; (2) age ≥ 18 years; (3) had clear thought processes; (4) gave informed consent to participate voluntarily; and (5) a course of disease ≥ 2 weeks and ≤ 6 months. The exclusion criteria were as follows: (1) patients with transient ischemic attack; (2) those with major organ failure; (3) those unable to communicate using words; and (4) those diagnosed with a mental disorder before experiencing a stroke.

A paper questionnaire was used for the study’s survey from October 2020 to May 2021. Prior to distributing the survey, the researcher communicated with the participants, answered their questions in detail, and guided them to complete it by themselves. Rehabilitation physicians uniformly assessed patients’ level of functioning and disability using the Barthel Index rating scale [47]. As the researcher guided the participants to fill in the questionnaire one-on-one, the recovery rate and effectiveness rate of the questionnaire reached 100%. The patients participated in this study voluntarily and did not receive any compensation for filling in the questionnaire. Participants signed written consent forms before data collection and the data collected are only available to researchers and the Ethics Review Committee. This article reports according to the STROBE checklist.

### Ethical consideration

The study was approved by the Ethics Committee of Shengjing Hospital of China medical university (approval number: 2020PS737K). The study conforms to Declaration of Helsinki.

### Measurements

#### Demographic data

Sociodemographic and disease-related data of patients with stroke were collected during the rehabilitation period, including patients’ gender, age, religious beliefs, marital status, residential area, educational level, medical insurance type, employment status, family per capita monthly income, stroke type, first or not first onset, and number of sequelae. The sequelae mainly included hemiplegia, speech disorder, sensory disorder, and swallowing disorder.

#### Psychological resilience

The Connor-Davidson Resilience Scale (CD-RISC), which was developed by Connor & Davidson [16], was used to measure the psychological resilience of patients with stroke. The Chinese version of CD-RISC has 25 items that are divided into three dimensions [48]: self-improvement (8 items), tenacity (13 items), and optimism (4 items). Each item is rated on a 5-point scale (0–4 points), and the total possible score ranges from 0 to 100. A higher score indicates greater psychological resilience. The internal consistency of the scale was 0.910, and Cronbach’s α for the three dimensions ranged from 0.600 to 0.880, and for the entire scale was 0.920. This instrument has acceptable concurrent validity; the total score correlates positively with hardiness (*r* = 0.83) and social support (*r* = 0.36) and negatively with perceived stress (*r* = -0.76) and stress vulnerability (*r* = -0.32).

#### Social support

Social support was measured using the Social Support Rating Scale (SSRS), which was developed by Xiao in 1994 [49]. The SSRS has 10 items and three dimensions: objective support, subjective support, and support utilization. Items 1–4 and 8–10 are rated on a 4-point scale. Item 5, ‘support and help from family members’, measures four possible levels of support ranging from 1 (no support) to 4 (full support), received from five categories of family members ranging from A (spouse) to E (other relatives). Items 6 and 7, which measure resources of support are scored as 0 points or 1–9 points, depending on the number of sources checked by the respondent. The total possible score ranges from 12 to 66 points, with a higher score indicating a higher the level of social support. The correlation coefficients between each scale and subscale are 0.360, 0.290 and 0.230. The correlation coefficients between the subscale and the total scale are 0.740, 0.850 and 0.760 [50]. In this study, Cronbach’s α for the SSRS was 0.789.

#### Hope

Hope was measured using the Herth Hope Index (HHI) [51], which consists of 12 items and three dimensions: a positive attitude towards reality and the future, taking positive action, and maintaining close relationships with others. The HHI is rated on a 4-point Likert-type scale ranging from 1 (completely disagree) to 4 (completely agree). Items 3 and 6 are reverse scored. The total score of the scale is the sum of the scores of all the items. The higher the score, the higher the respondent’s level of hope. All 12 items had a significant loading on one of the three factors as was originally formed subscales of the HHS. Divergent validity was assessed by calculating the correlation of the HHI to the Hopelessness Scale (*r* = -0.73). In this study, Cronbach’s α for the HHI was 0.820.

#### Self-esteem

Self-esteem was measured using Rosenberg’s Self-Esteem Scale (SES), which was developed by Rosenberg [52]. The SES consists of 10 statements focusing on general feelings toward oneself. Participants are asked to report their level of agreement with statements on a 4-point Likert scale ranging from 1 (agree - not at all) to 4 (agree - completely) for Items 1, 2, 4, 6, 7, and 8. Items 3, 5, 9, and 10 are reverse scored, and a higher total score indicates a higher degree of self-esteem. The SES is the most widely used instrument for estimating levels of self-esteem, and it has high levels of reliability and validity [53]. The test-retest reliability of the SES was 0.850, and, in this study, Cronbach’s α was 0.790.

### Data analysis

SPSS 26.0 (IBM Corp, Armonk, NY) was used for the statistical analyses. Pearson’s correlation coefficient was used to compare correlations between the four variables of interest. Hierarchical regression analysis was used to examine the factors influencing patients’ resilience. The collinearity between variables was diagnosed before hierarchical regression analysis. Amos 26.0 (IBM Corp, Armonk, NY) was used to conduct structural equation modeling, with social support and self-esteem as the exogenous independent variables, hope as the mediating variable, and resilience as the dependent variable. The maximum likelihood method was used. The overall fitness indexes of the model should be as follows: GFI, IFI, CFI, and TLI > 0.9; and RMSEA < 0.08, CMIN/df < 3, and SRMR < 0.08 [53, 54]. When a 95% confidence interval did not include 0, the indirect effect (mediation) was considered statistically significant; *P* < 0.05 was considered statistically significant.

## Results

### Characteristics of the participants

A total of 210 valid questionnaires were analysed. Women accounted for 38.8% of all respondents; patients aged 18–44 years accounted for 18.8%; those aged 45–59 years accounted for 39.4%; and those older than 60 years accounted for 41.9%. The mean resilience score of the patients was 59.88 ± 16.11, and the mean social support score was 36.17 ± 7.99. The mean hope score was 35.78 ± 5.58 and the mean self-esteem score was 75.77 ± 19.60 Patients’ scores on all of the dimensions of the variables of interest are shown in Table 1.

**Table 1:** The score of resilience, social support, hope and self-esteem of stroke patients in rehabilitation stage

Variables	Score range	Score(M ± SD)
Resilience		
Tenacity	8 ~ 49	28.99 ± 9.34
Self-improvement	6 ~ 31	21.18 ± 5.27
Optimism	1 ~ 19	9.23 ± 3.08
Total score	15 ~ 92	59.88 ± 16.11
Social support		
Objective support	3 ~ 18	9.71 ± 2.82
Subjective support	7 ~ 32	19.08 ± 6.23
Support utilization	3 ~ 14	7.33 ± 2.11
Total score	19 ~ 56	36.17 ± 7.99
Hope		
Positive attitudes towards reality and the future	7 ~ 16	11.84 ± 2.07
Taking positive actions	7 ~ 16	12.14 ± 1.82
Maintaining close relationships with others	6 ~ 16	11.85 ± 2.22
Total score	22 ~ 48	35.78 ± 5.58
Self-esteem	17 ~ 37	28.61 ± 4.31

### The relationships between social support, self-esteem, hope, and resilience

Pearson correlations showed that the scores for social support, positive attitude, positive action, intimate relationship, total hope, and self-esteem were positively correlated with the total and dimension score for psychological resilience (all *Ps* < 0.010), which supported *Hypothesis* 1 and 2. See Table 2 for details.

**Table 2:** Correlation Analysis between resilience and other variables of stroke patients in rehabilitation stage

Variables	Tenacity	Self-improvement	Optimism	Total score
Social support				
Objective support	0.153	0.329**	0.284**	0.254**
Subjective support	0.479**	0.345**	0.449**	0.459**
Support utilization	0.121	0.236**	0.219**	0.182*
Total score	0.47**	0.457**	0.518**	0.507**
Hope				
Positive attitudes towards reality and the future	0.671**	0.545**	0.544**	0.666**
Taking positive actions	0.614**	0.442**	0.447**	0.587**
Maintaining close relationships with others	0.630**	0.521**	0.540**	0.637**
Total score	0.719**	0.567**	0.578**	0.711**
Self-esteem	0.608**	0.610**	0.566**	0.671**

**P＜0.01;*P＜0.05

### Results of the hierarchical regression analysis

Hierarchical regression analysis was carried out with the total score of psychological resilience as the dependent variable and the variables that have a significant impact on psychological resilience in socio-demography, social support, self-esteem and hope as the independent variables. The variance inflation factor of each variable entering the regression model is less than 10, except marital status. There are two eigenvalues less than 0.01, two condition indexes greater than 30, and the maximum condition index is 43.537, indicating that there may be a weak collinearity problem between independent variables. From the perspective of variance proportions, there was no variance proportions of two independent variables on a certain eigenvalue greater than 0.7, indicating that the linear coincidence between independent variables is not serious. Therefore, there is no serious multicollinearity problem after the respective variables enter the regression model (see *Appendix 1* for the results of collinearity diagnostics).

The results of the hierarchical regression showed that the overall model had a good fit (*P* < 0.001). When hope was not included in the model, social support, self-esteem had a significant impact on resilience. When hope was included as an independent variable, the magnitude of the associations of social support and self-esteem with resilience decreased (see Table 3).

**Table 3:** Hierarchical regression analysis results

Independent variables		B	SE	β	t	P
*First stage (Adjusted R*^*2*^ *= 0.524, F = 14.488, p < 0.001)*						
	Constant	-2.662	12.138		-0.219	0.817
	Religious belief	1.537	2.882	0.031	0.533	0.595
Marital status	Unmarried	-5.954	8.571	-0.098	-0.695	0.488
	Married	-10.995	7.904	-0.286	-1.391	0.166
	Divorce	-15.194	8.560	-0.258	-1.775	0.078
	Widowed	-7.338	5.939	-0.153	-1.236	0.219
Educational level	College degree or above	1.884	2.247	0.057	0.839	0.403
	Primary school and below	-6.022	3.727	-0.099	-1.616	0.108
Family per capita monthly income (yuan)	< 1500	0.217	2.800	0.006	0.077	0.938
	1500 ~ 3000	-0.678	2.296	-0.020	-0.295	0.768
Number of sequelae	No	18.557	5.802	0.180	3.198	0.002
	One kind	1.263	1.928	0.039	0.655	0.513
	Social support	0.449	0.134	0.223	3.352	0.001
	Self-esteem	2.086	0.249	0.558	8.394	< 0.001
*Second stage (Adjusted R*^*2*^ *= 0.598, F = 17.926, p < 0.001)*						
	Constant	-16.694	11.465		-1.456	0.148
	Religious belief	2.528	2.655	0.051	0.952	0.343
Marital status	Unmarried	-9.418	7.903	-0.154	-1.192	0.235
	Married	-12.823	7.271	-0.333	-1.764	0.080
	Divorce	-16.230	7.868	-0.276	-2.063	0.041
	Widowed	-5.422	5.469	-0.113	-0.991	0.323
Educational level	College degree or above	-3.927	3.447	-0.064	-1.139	0.257
	Primary school and below	3.102	2.078	0.094	1.493	0.138
Family per capita monthly income (yuan)	< 1500	1.788	2.590	0.046	0.690	0.491
	1500 ~ 3000	0.321	2.119	0.010	0.151	0.880
Number of sequelae	No	15.067	5.372	0.146	2.804	0.006
	One kind	1.540	1.773	0.048	0.869	0.387
	Social support	0.292	0.135	0.145	2.171	0.032
	Self-esteem	0.989	0.283	0.264	3.496	0.001
	Hope	1.199	0.227	0.416	5.283	< 0.001

### Hope mediates the relationships of social support and self-esteem with resilience

The demographic variables with statistical significance in hierarchical regression analysis were used as confounding variables, that is divorce and sequelae. The overall fitness indexes of the structural equation model were CMIN/df = 1.880, RMSEA = 0.074, GFI = 0.958, IFI = 0.959, CFI = 0.958, TLI = 0.936, and SRMR = 0.061. They showed that the model had a good fit overall and the standardized path was as shown in Fig. 1. After controlling for divorce and sequelae variables, hope mediated the relationships between social support, self-esteem, and resilience. A positive relationship was found between social support and resilience (*β1* = 0.548, 95% CI [0.219, 0.613]), which was mediated by hope (*β2* = 0.114, 95% CI [0.050, 0.286]); social support had significant direct effect on resilience (*β3* = 0.434, 95% CI [0.320, 0.693]). The results supported *Hypothesis3*. A positive relationship was found between self-esteem and resilience (*β4* = 0.380, 95% CI [0.225, 0.577]), which was mediated by hope (*β5* = 0.200, 95% CI [0.141, 0.622]), and self-esteem had significant direct effect on resilience (*β6* = 0.179, 95% CI [0.035, 0.328]). The results supported *Hypothesis4*. See Table 4 for details. The hope partially mediated the relationship between social support/self-esteem and resilience in individuals after stroke.

**Table 4:** Total effects and indirect effects among variables (*N* = 210) SE: Standard error

	B	β	SE	95%CI	P
Total effects					
Social support →Hope	0.584	0.315	0.108	(0.099, 0.392)	< 0.001
Social support →Resilience	4.360	0.548	0.135	(0.219, 0.613)	0.014
Self-esteem→Hope	0.236	0.550	0.087	(0.419, 0.763)	0.001
Self-esteem →Resilience	0.699	0.380	0.126	(0.225, 0.577)	0.016
Hope→Resilience	2.350	0.360	0.145	(0.250, 0.856)	0.003
***Direct effects***					
Social support →Resilience	3.448	0.434	0.139	(0.320, 0.697)	0.008
Self-esteem →Resilience	0.330	0.179	0.137	(0.035, 0.328)	0.033
***Indirect effects***					
Social support→ Hope → Resilience	0.912	0.114	0.047	(0.050, 0.286)	< 0.001
Self-esteem → Hope → Resilience	0.369	0.200	0.094	(0.141, 0.622)	0.001

**Fig. 2:** Final model and standardized model paths

## Discussion

### Current status of psychological resilience

The level of psychological resilience of patients with stroke during the early rehabilitation stage in this study (52.43 to 62.19) was lower compared to healthy populations in other studies [16], which supports the need to help patients after a stroke improve their psychological resilience.

The results of this study show that the psychological resilience score of stroke individuals with religious beliefs was higher, which is consistent with the results in other affected populations, such as breast cancer patients [55] and people who have experienced trauma or stressful events [56]. The psychological resilience of divorced individuals with stroke was worse, which can be explained by the fact that the relationship between husband and wife is a key factor affecting the level of psychological resilience of patients with chronic diseases [57]. Individuals with high monthly income showed better psychological resilience because of the lower economic burden and the coping obstacles in the face of such frustrating events. Stroke patients with high education have a higher level of psychological resilience. Educational intervention also played a positive role in reducing helplessness and discomfort in other studies [58]. Therefore, during hospitalization, health providers should regularly popularize disease-related knowledge for stroke convalescent patients so that patients can become deeply familiar with the reason and treatment of stroke, which will help patients better understand the disease and receive treatment in the hospital, community, and family. Furthermore, the more sequelae, the lower the level of psychological resilience of stroke patients. The sequelae of stroke, such as hemiplegia, speech inability, sensory, and swallowing disorders, can bring great psychological pressure to patients, resulting in lower psychological resilience.

The above results on the influencing factors in the general characteristics of psychological resilience of stroke patients were basically consistent with other studies in patients with stroke. What caregivers can do is to use different focus care methods according to different characteristics of patients. Appropriate intervention and treatment measures are also needed to reduce the sequelae of stroke. At the same time, the author also found that the research on psychological resilience of stroke patients is relatively small. Considering the important role of psychological resilience in post-stroke depression and the characteristics of post-stroke depression, it is necessary to strengthen research on psychological resilience in the early rehabilitation after stroke.

### The mediating role of hope in the relationships of social support and self-esteem with psychological resilience

Research shows that the first 6 months after a stroke are the period of physical and mental recovery [59]. Psychological resilience is an independent predictor of post-stroke depression and quality of life [60], and post-stroke depression can be alleviated by improving psychological resilience [61]. Using a cross-sectional survey, this study explored the roles of social support, self-esteem, and hope as predictors of psychological resilience in patients with stroke. This study found that social support and self-esteem were predictors of psychological resilience. When hope was included in a model of the relationship between social support and self-esteem with psychological resilience, the direct effects of social support and self-esteem were reduced, due to the mediating effect of hope.

The social support of patients with stroke during the early rehabilitation stage can indirectly affect their resilience levels, which is consistent with the results of other studies: A study of patients with breast cancer undergoing treatment found that hope played a complete mediating role between social support and resilience [62]. A study on patients with prostate cancer also showed that hope played a mediating role in the relationship between social support and psychological state [63]. Perceived social support can improve an individual’s overall level of happiness and promote the establishment of positive qualities, including hope [64]. The construction of hope is closely related to perceived social support [65]. According to Snyder’s theory of hope, perceived social support is an important factor affecting hope. For example, perceived social support from parents and friends is beneficial for the establishment and development of hope [66, 67]. Previous studies have also found a significant positive correlation between social support and hope [68]. There is also a connection between hope and resilience. Ong et al. [69] believed that hope may be one of the important sources of psychological resilience. Hope can not only reduce negative emotions and protect individuals but also help promote social adaptation and recovery from stress. Empirical research has confirmed a significant positive correlation between hope and resilience [70, 71]. Additionally, previous studies have found that hope can significantly and positively predict resilience [72], and hope may be an important factor in promoting resilience [73]. Condly’s review of psychological research on children and resilience suggests that adults with resilience typically attribute their resilience as children to hope [74]. Therefore, it was assumed by previous researchers that perceived social support may also affect psychological resilience through hope, which is proved by this study.

This indirect effect may be because patients with high social support receive more iatrogenic support and support from surrounding people. The encouragement and company of others enhance patients’ confidence in recovery from their disease, enable them to cooperate actively with the treatments and procedures of medical personnel, help them regain hope in their recovery, and increase their level of resilience [60]. Social support is an important protective factor against stressful events, and protective factors are necessary for the recovery process [22]. Therefore, when treating and caring for patients during the early stage of stroke rehabilitation, medical staff should also pay attention to the patient’s level of hope in their recovery; guide patients in affirming their own value, and encourage them to evaluate their own shortcomings, perceived threats, and fears precipitated by the stroke.

The present study’s results showed that patients’ self-esteem during the early rehabilitation stage after a stroke can indirectly affect their level of resilience. A study of patients with severe mental illness showed that hope mediated the relationship between self-esteem and quality of life [75]. Another study found a moderate association between hope and self-esteem (*r* = 0.49, *P* < 0 0.001) among people in the early stages of dementia [76] and concluded that self-esteem affects a person’s hope for the future. However, hope was found to be a predictor of self-esteem, which is contrary to our study’s results and the results of the study by Mashiach-Eizenberg et al. [75]. Hence, there is no clear theoretical or empirical evidence for a causal relationship between self-esteem and hope, which is a research direction for the future.

### Implicate the findings into nursing practice

Many interventions can be used to enhance the psychological resilience of the elderly, such as oral encouragement to enhance self-efficacy, build self-esteem, maintain optimism, and establish positive interpersonal relationships. However, the experience of stroke makes the implementation of these types of interventions challenging. Overcoming these challenges and enhancing individual psychological resilience after stroke is very important for individual rehabilitation. Psychological resilience gives individuals the strength to recover from adversity. According to the results of this study, some strategies can be incorporated into the rehabilitation process to enhance psychological resilience: (1) cultivate individual personality characteristics, such as hope, optimism, self-esteem, etc.; (2) Improve patients’ social relationships, such as social support. First, the key to remaining optimistic after a stroke is related to retaining the element of hope: helping stroke patients see progress in their goals, continue their potential rehabilitation, and build faith in a valuable and productive future. Secondly, in addition to health education for family members and enhancing patients’ social support, patients can also be encouraged to join social groups, exercise, or participate in voluntary activities, and mobilize their self-care and self-management ability. Additionally, it is recommended that future studies use longitudinal study design or experimental study design to further analyze the mediating effect between variables to clarify the causal relationship and improve the credibility and power of the research results.

### Limitations

First, this cross-sectional study investigated only the level of psychological resilience of patients with stroke during the early stroke rehabilitation stage; however, psychological resilience is a dynamic process. We should investigate the level of psychological resilience of patients with stroke in different stages of the illness (i.e., the acute, recovery, and sequelae stages), and explore the status and the factors influencing the level of psychological resilience in in the different stages. Second, the Psychological Resilience Scale currently used is a universal scale. The specificity of the information yielded on the psychological resilience of patients with stroke in the convalescent stage needs to be improved. Developing a psychological resilience scale suitable for this population is a necessary research direction, which should provide a reference for the prevention of, and solutions for psychological distress among patients with stroke and for implementing mental-health nursing interventions. Third, we explored the protective factors of psychological resilience, and the Multi-System Model of Resilience proposed by Liu, Reed, & Fung [77] showed that psychological resilience is also affected by risk factors (such as exposure to stress and adversity). Therefore, we need to explore methods for improving psychological resilience among patients with stroke in combination with their risk factors to improve their quality of life and reduce the incidence of post-stroke depression. Fourth, this study is a cross-sectional study, which hinders the causal inference between variables. In the future, longitudinal study design or experimental study can be considered to verify the cross-sectional study results and better explore the causal relationship. Therefore, the current cross-sectional study can provide preliminary support for the mediation process described. Finally, there are communalities in what is measured in resilience, social support and hope scales, given that resilience and social support are measured by the Hope scale to some extent. In the future, study should carefully examine the specific items within each scale to identify any potential redundancies or shared variance among the constructs, and provide a more comprehensive discussion on the potential interrelations among resilience, social support, and hope, highlighting the nuances and complexities of these constructs.

## Conclusion

Despite some limitations, this study provides preliminary support for explaining and elucidating the mediating role of hope in the relationship between social support, self-esteem, and psychological resilience in in patients with stroke during the early rehabilitation stage. Psychological resilience is very important for improving a patients’ quality of life and alleviating post-stroke depression. Therefore, in future studies, the personality characteristics of patients with stroke should be evaluated as soon as possible to predict their level of psychological resilience and improve their social support system, as indicated during early stroke rehabilitation.

### Electronic supplementary material

Below is the link to the electronic supplementary material.

Supplementary Material 1: The results of collinearity diagnostics

## Data Availability

The datasets used and/or analysed during the current study are available from the corresponding author on reasonable request. The author confirmed that we didn’t use AI tools to analyse and draw insights from data as part of the research process. This manuscript has not been published or presented elsewhere in part or entirety and is not under consideration by another journal.
